The article "Risk prediction of gestational diabetes mellitus in women with polycystic ovary syndrome based on a nomogram model" was published in 2023. Journal: BMC Pregnancy Childbirth.

# Risk prediction of gestational diabetes mellitus in women with polycystic ovary syndrome based on a nomogram model

**DOI:** 10.1186/s12884-023-05670-x

**Published:** 2023-06-02

**Authors:** Peilin Ouyang, Siqi Duan, Yiping You, Xiaozhou Jia, Liqin Yang

**Affiliations:** Hunan Provincial Maternal and Child Health Care Hospital, 53, Xiangchun Road, Changsha, Hunan People’s Republic of China

**Keywords:** Polycystic ovary syndrome, Gestational diabetes mellitus, Nomogram model

## Abstract

Women with polycystic ovary syndrome are prone to develop gestational diabetes mellitus, a disease which may have significant impact on the postpartum health of both mother and infant. We performed a retrospective cohort study to develop and test a model that could predict gestational diabetes mellitus in the first trimester in women with polycystic ovary syndrome. Our study included 434 pregnant women who were referred to the obstetrics department between December 2017 and March 2020 with a diagnosis of polycystic ovary syndrome. Of these women, 104 were diagnosed with gestational diabetes mellitus in the second trimester. Univariate analysis revealed that in the first trimester, Hemoglobin A1c (HbA1C), age, total cholesterol(TC), low-density lipoprotein cholesterol (LDL-C), SBP (systolic blood pressure), family history, body mass index (BMI), and testosterone were predictive factors of gestational diabetes mellitus (*P* < 0.05). Logistic regression revealed that TC, age, HbA1C, BMI and family history were independent risk factors for gestational diabetes mellitus. The area under the ROC curve of the gestational diabetes mellitus risk prediction model was 0.937 in this retrospective analysis, demonstrating a great discriminatory ability. The sensitivity and specificity of the prediction model were 0.833 and 0.923, respectively. The Hosmer–Lemeshow test also showed that the model was well calibrated.

## Introduction

Gestational diabetes mellitus (GDM) is defined as glucose intolerance that develops or is first diagnosed during pregnancy after the first trimester of pregnancy and is not caused by type 1 or type 2 diabetes mellitus [1].GDM has long-lasting harmful effects on both the mother and infant [2]. Women with a history of GDM are almost ten times more likely to develop type 2 diabetes mellitus than those without [3]. Maternal hyperglycemia may also place offspring at risk of autism spectrum disorders, obesity, hypertension, type 2 diabetes, hyperlipidemia, cardiovascular disease [4, 5].

The global incidence of GDM ranges from 9 to 25%, while in China it ranges from 13.0% to 20.9% [6]. The increasing incidence of GDM is likely to associated with a greater rate of maternal obesity and a trend of lowering diagnostic criteria [7, 8].

Over the last 10 years, the incidence in our hospital has been risen from 13.4% to 16.3%. Polycystic ovary syndrome (PCOS) is a common disorder that affects 8% of reproductive-aged women [9, 10]. The syndrome is also associated with various comorbidities that cause obesity, and have long-term sequelae such as insulin resistance and metabolic syndrome [11]. Women with PCOS have higher levels of insulin resistance, which predisposes them to developing GDM [12]. Based on extensive clinical research, the National Institutes of Health reported that PCOS is an independent risk factor for GDM. PCOS has become the most common endocrine and gynecological condition in Chinese women of childbearing age because of a shift from a traditional Chinese diet to a high-sugar, high-fat diet, and a delayed childbearing age [13].

Therefore, it is critical to identify pregnant women with PCOS who are at risk of developing GDM. The objective of this study was to eastablish an early predictive, model of GDM for women with PCOS,and may provide early intervention measures to benefit patients.

## Patients and methods

### Inclusion and exclusion criteria for patients

This retrospective cohort study used data from the medical records of 434 women with PCOS. The patients were between 7 and 12 weeks pregnant and have prenatal examinations in the Hunan Provincial Maternal and Child Health Care Hospital between December 2017 and March 2020. Follow-up was performed regularly. Patients were included if they 1) were pregnant and had PCOS; 2) were older than 18 years; 3) intended to have prenatal examinations and deliver their infants at our hospital; and 4) had an oral glucose tolerance test at 24–28 weeks of pregnancy. Patients were excluded if they had 1) pregestational diabetes mellitus or diagnosed as gestational diabetes in the first trimester; 2) cardiovascular, respiratory, thyroid, liver, kidney, or any other diseases that might affect the research outcomes.

The diagnosis of PCOS was based on the Rotterdam criteria. It is characterized by the presence of at least two of the following diagnostic criteria: 1) hyperandrogenism and/or biochemical signs of hyperandrogenism; 2) polycystic ovaries determined sonographically with 12 or more measured follicles of length between 2 and 9 mm; 3) ovulatory dysfunction (oligo-ovulation or anovulation) [11].

## Data collection

Plasma samples and general information were collected from all participants at the first clinical visit in the first trimester ( 7–12 gestational weeks). Standard sphygmomanometry was used to measure blood pressure in each patient. The measurement unit of Weight and Height were recorded and rounded to the nearest 0.1 kg and 0.1 cm, respectively. BMI was counted by dividing the weight by the square of height. Patients with a BMI of between 24.0 and 27.9 kg/m^2^ were defined as “overweight”, while those with a BMI of more than 28.0 kg/m^2^ were defined as “obese” [14]. After an 8 h overnight fasting period in the morning, venous blood samples were collected. TG, TC, high-density lipoprotein cholesterol (HDL-C), low-density lipoprotein cholesterol (LDL-C), FBG, HbA1C and testosterone levels were measured.. All the samples were sent at once to the Laboratory of the Hunan Provincial Maternal and Child Health Care Hospital for testing. Laboratory biochemical indicators were measured using an Olympus AU2700 biochemical analyzer (Olympus Corp).

## GDM diagnosis

GDM was screened for by performing an oral glucose tolerance test on patients during weeks 24–28 of pregnancy: patients included in the study fasted for 8 to 12 h overnight, and the following morning drank 250–300 mL water with 75 g glucose powder dissolved and drunk within 5 min. Their venous blood was measured before the examination, and then again after 1 and 2 h. The diagnostic standard used for gestational diabetes was that of abid by the International Association of Diabetes and Pregnancy Study Group (IADPSG) [15]. Patients were diagnosed with GDM if they blood glucose level reached any one of it: fasting blood glucose level ≥ 5.1 mmol/L, blood glucose at 1 h after glucose intake ≥ 10.0 mmol/L, or blood glucose at 2 h after glucose intake ≥ 8.5 mmol/L.

## Statistical analysis

Descriptive statistic analyses were performed to analysis 434 participants using IBM SPSS Statistics for Windows, Version 20.0 (Armonk, NY: IBM Corp.). Non-normally distributed continuous variables were presented as medians (interquartile ranges), while normally distributed data were presented as means ± standard deviations. Categorical variables were expressed as frequency (n) and proportions (%). The chi-square or Fishers exact test was used to analyze categorical variables. T-test or Wilcoxon test was used to analyze continuous variables.

The nomogram model was developed and implemented in three steps. First, using nonzero coefficients in the least absolute shrinkage and selection operator (LASSO) regression model, we identified independent predictive features [16]. Second, the selected variate from the LASSO regression model were identified to construct the multivariate logistic regression model, and selected the variables with statistical significance to establish the nomogram model [17]. Third, the nomogram’s discrimination and calibration were evaluated using calibration curve plots, the area under the receiver (AUC), and Harrell’s concordance index (C-index), respectively, and K-fold cross-validation was used (k = 10) to validate the model. All Figures were created using R software, version 4.1.1; the glmnet-package and matrix-packages were used to realize LASSO, and a regression-nomogram model were built using the R packages ‘*lattice*,’ ‘*Formula*,’ ‘ggplot2,’ ‘survival,’ and ‘rms.’ And the R-package. Nomogram EX was used to convert the nomograms into equations, and ROC curves were run with the pROC-package. (http://www.R-project.org).

## Results

### Baseline characteristics

The study cohort comprised 434 women, among whom 104 were diagnosed with GDM during the second trimester(30.3%). The average age of the GDM patients was 29 years, the proportion of patients with age ≥ 35 years old was no significant difference between the two groups.The GDM patients also exhibited relatively elevated levels of BMI, TG, TC, FPG, LDL, testosterone and HbA1c%, as well as a higher prevalence of family history of diabetes (*p* < 0.05). However, there were no statistically significant differences in blood pressure and HDL levels between the two groups (Table 1).

**Table 1:** Comparison of first trimester laboratory test and general conditions of PCOS women between the GDM and non-GDM groups

Variable	GDM group (*n* = 104)	Non-GDM group (*n* = 330)	*P*-value
**Age(years)**			
< 35	94(90.4%)	307(93.0%)	0.433
≥ 35	10(9.6%)	23(7.0%)	
**BMI(kg/m2)**			
< 24	51(49.0%)	301(91.2%)	P < 0.05
24 ≤ n < 28	51(49.0%)	29(8.8%)	
≥ 28	2(2.0%)	0(0.0%)	
**Parity**			
0	57(54.8%)	244(73.9%)	P < 0.05
≥ 1	47(45.2%)	86(26.1%)	
**Family history with diabetes**			
No	75(72.1%)	313(94.8%)	P < 0.05
Yes	29(27.9%)	17(5.2%)	
**Testosterone (mmol/L)**	1.28(0.77,1.71)	1.48(0.92,1.99)	0.022
**LDL(mmol/L)**	2.92(1.16,3.34)	1.62(1.00,2.08)	0.000
**HDL(mmol/L)**	1.19(1.01,1.46)	1.09(0.85,1.50)	0.120
**TG(mmol/L)**	2.29(1.51,3.05)	1.54(1.02,2.17)	0.000
**TC(mmol/L)**	4.81(4.32,5.17)	3.24(2.32,3.92)	0.000
**FPG(mmol/L)**	4.42 ± 0.42	4.42 ± 0.36	0.000
**HbA1c(%)**	5.08 ± 0.47	4.64(4.37,4.93)	0.000
**SBP(mmHg)**	117(112,125)	118(112,123)	0.560
**DBP(mmHg)**	75(68,81)	75(69,82)	0.477

*MI* Body mass index, *SBP* Systolic blood pressure, *DBP* Diastolic blood pressure, *FPG* Fasting plasma glucose, *HbA1c* Glycosylated hemoglobin, *TC* Total cholesterol, *TG* Triglycerides, *LDL-C* Low-density lipoprotein cholesterol, *HDL-C* High-density lipoprotein cholesterol

### Univariate and multivariate analysis

The feature selection was used for the LASSO, which appears to be a strong rival for variable selection in the Cox model [18]. LASSO regression analysis minimizes the prediction error of quantitative response variables by imposing constraints on model parameters that cause the regression coefficients of some variables to shrink to zero. Variables with zero regression coefficients after the contraction process were excluded from the model, while variables with non-zero regression coefficients had the strongest correlation with response variables. The method selected eight optimal predictors for the regression model, including HbA1C, age, TC, LDL-C, SBP, family history, BMI, and testosterone. Then, eight variables were used to construct the multivariate logistic regression model Fig. 1.

**Fig. 1:** **a** The Feature selection was used for the least absolute shrinkage and selection operator (LASSO). An optimal parameter (lambda) was selected using minimum criteria according to tenfold cross-validation in the LASSO model. LASSO coefficient profiles of the 13 features. A coefficient profile plot was produced against the log (lambda) sequence. **b** A vertical line was drawn at the value selected using tenfold cross-validation, where optimal lambda resulted in 8 features with non-zero coefficients.

According to the multivariate logistic regression model, we defined the independent risk factors for GDM to include BMI (OR: 1.561; 95%CI: 1.315–1.882), HbA1C (OR: 7.770; 95%CI: 3.675–17.475), age (OR: 1.153; 95%CI: 1.039–1.287), TC (OR: 2.696; 95%CI:1.751–4.309), and family history (OR: 3.569; 95%CI: 1.408–9.440) (Table 2). Ultimately, the prediction model was built using five variables with *P*-values less than 0.05 in multivariate regression analysis (Table 2).

**Table 2:** GDM risk factors according to Multivariate logistic analysis

	β Coefficient	Wald test	*P*	OR(95%CI)
HbA1C	2.050	5.173	0.000	7.770 (3.675–17.475)
TC	0.992	4.341	0.000	2.696 (1.751–4.309)
BMI	0.445	4.899	0.000	1.561 (1.315–1.882)
Family history	1.272	2.636	0.008	3.569 (1.408–9.440)
Age	0.142	2.630	0.008	1.153 (1.039–1.287)

*HbA1c* Glycosylated hemoglobin, *TC* Total cholesterol *BMI* Body mass index

### Nomogram and evaluation of prediction model for gestational diabetes mellitus

The corresponding score of each predictor was displayed in the nomogram model (Fig. 2), and each variable can be quantified by drawing a vertical line straight to the point axis. The total score in the nomogram model was obtained by summing the individual item scores. We used the R package “nomogram EX” to convert the nomogram into the following Eq. (36.81418202 * HbA1C – 132.531055273) + (2.472388155* Age – 49.447763106) + (15.961470412* TC- 23.942205618) + (7.142857143* BMI – 114.285714286) + (23.31008* Family history). The probability of GDM was calculated as: Risk of GDM = -8.06e-07 * points ^3 + 0.000435015* points ^2 + -0.066933226 * points + 3.151391273. For example, in a 26-year old pregnant woman in the first trimester with a family history of diabetes, the BMI is 21 kg/cm^2^, serum cholesterol of 3 mmol/L, and serum HbA1c level of 4.8%, the total score was calculated as 142 with a corresponding probability of 11% for GDM during pregnancy.

**Fig. 2:** GDM nomogram for the first trimester. The risk of predicting the occurrence of GDM is quantified as the number of points marked on the axis, the score determined by each variable axis is the number corresponding to the value vertical on the total points scale, and projected the sum of all variables onto the bottom axis, yielding a personalized GDM risk for each woman with PCOS

Figure 3 shows the predictive performance of the model. The AUC of the ROC curve was 0.937. 0.186 (0.833, 0.923) is the best cult off value in the ROC curve, which means When the risk probability is 0.186 as the cutoff point, the sum of the sensitivity and specificity of the prediction result is the largest, was 83.3% and 92.3% respectively. The calibration of the prediction model was evaluated using the Hosmer–Lemeshow goodness of fit test, and a calibration curve was obtained, which showed good agreement to predict the GDM risk in first-trimester pregnant women with PCOS. K-fold cross-validation was used (k = 10) to validate the model, and the mean value of ten-fold cross-validation was 0.903 for AUC, 0.522 for R^2^ (coefficient of determination), and 0.418 for discrimination index, indicating well callibrated and strong classification ability of the model.

**Fig. 3:** **a** The ROC curves showing the precision of the GDM nomogram in patients. The AUC of the nomogram was 0.937, when the risk probability is 0.186 as the cutoff point,the validation model’s sensitivity and specificity were 0.833 and 0.923, respectively. **b** The y-axis represent the actual diagnosed GDM. The x-axis represent the predicted risk of GDM. The dotted diagonal line represent a perfect prediction by an ideal model. The predict curve showed a closer fit to the dotted diagonal line represented the model was well calibrated

## Discussion

GDM has many effects on both pregnancy outcomes and long-term neonatal complications. Several predictive models for GDM have been developed by integrating patients' general characteristics, clinical test results, genetic information, and other relevant data. Sirico et al. demonstrated that higher fetal heart rates (FHR) in the first trimester were an independent risk factor for GDM [19]. This finding was further confirmed in a multicenter study, where an FHR threshold of 162 bpm showed a detection rate of 76.9%, specificity of 67.1%, and negative predictive value of 85.5% for GDM [20].Sweeting et al. constructed a multivariate prediction model that combined clinical risk factors with novel biomarkers, including PAPP-A, triglycerides, and lipocalin-2, which accurately predicted GDM in early pregnancy with an area under the curve of 0.93 (95% CI 0.89–0.96) for early GDM [21].PCOS is a risk factor for GDM and was confirmed in a study by Weerakiet S more than 10 years ago [1]. The same validation was obtained in the study by Toulis KA [2]. A meta-analysis performed by Jing Z found that the incidence of GDM was reduced by using metformin, suggesting that metformin is effective for preventing GDM in PCOS patients. Therefore, the risk factors for GDM in PCOS women can guide clinicians to early prevention and intervention to reduce occurrence [3]. In our study, we combined five independent risk factors, including BMI, HbA1C, age, TC, and family history, to construct a nomogram model to predict the risk of GDM in women with PCOS in their first trimester.

Type 2 diabetes exhibits insulin resistance and elevated blood glucose levels, which may promote pathological harm in PCOS patients [22]. It is generally accepted that Fatty acids(FAs) play a major role in the development of insulin resistance [23]. In our study, TC is the positive index to indicate the occurrence of GDM in pregnant women with PCOS. Several studies have reported that dyslipidemia in the first trimester of pregnancy is related to the development of GDM [24, 25]. Lean or obese women with higher TG concentrations have an increased risk of developing GDM, whereas lean women with high HDL-C levels do not. This statement is consistent with O’Malley, who stated that maternal obesity mediates the epidemiological relationship between GDM and dyslipidemia, and only women with GDM who were obese had higher TG and lower HDL-C levels and a higher TG: HDL-C ratio than those without GDM [26]. A retrospective study indicated that women with GDM are more likely to have hyperlipidemia postpartum, particularly dyslipidemia defined by TG [27]. Hyperinsulinemia is usually concomitant with low HDL cholesterol and high LDL–cholesterol levels. The increased release of free fatty acids from insulin-resistant fat cells may be the cause of these characteristics [28]. Dyslipidemia, which is associated with diabetes mellitus, is the main risk factor for the development of cardiovascular disease. Diabetes-related lipid changes are attributed to an increased free fatty acid flux caused by insulin resistance. However, the varies of TG was not included in our nomogram model, it may attributed to the different value units and classification of grading methods.

HbA1c is also an indicator for Abnormal glucose regulation, to enable early recognition and intervention of GDM. Based on the prospective analysis for 1,989 pregnant women, Yi-Ran Ho etc. conluded that the when the level of HbA1c achive to 5.7%, the AUC(Area Under The Curve) of the ROC curvce was 0.70 and significantly associated with increased risks of neonatal complications like neonatal intensive care unit, low birth weight, and macrosomia [29]. Burke Schaible etc. showed that HbA1C also was a reliable indicator to GDM for pregnant women in first trimester. They included 146 patients and recommended that an HbA1c threshold of 5.15% can identify 66.7% of pregnant women with abnormal oral glucose tolerance test at 24–28 weeks [30]. While, a large cohort study in China demonstrated that the HbA1c test offers limited value in GDM diagnoses. A total of 19,261 pregnant were enrolled in this study, and Yi Lai et al. found that level of HbA1c is 5.0% as the cutoff point, the sensitivity and specificity was 60.1% and 65.3% respectively. It maybe attributed that the HbA1 level changes is delayed to identify certain cardiometabolic changes. In our study, logistic regression result shows that the level of HbA1c is the significant factor to predict GDM. Consequently, it would be useful to have a clinical index that could quantify the differences between women with PCOS who have GDM and those who do not have. It was shown that both insulin sensitivity and β-cell function are significantly decreased with a 0.6% increase in glycohemoglobin and that insulin resistance can be found by detecting HbA1C [13].

In our study, BMI is the significant index to indicate the occurrence of GDM in pregnant women with PCOS. N.S. Kakoly pointed out that obese women with PCOS patients are more likely to develop insulin resistance or type 2 diabetes mellitus later, and this results were independent of race [31]. According to previous studies, the most important risk factor for GDM is being overweight or obese prior to pregnancy (BMI 25 kg/m^2^ or above) [32]. This was not affected by the geographical distribution, parity, or a history of GDM. However, a previously reported clinical model that used BMI as the independent factor to screen for GDM found that the outcomes varied widely by race: GDM was found in more than 76% of African-Americans, 58% of Latinas, and 46% of Caucasians, but only 25% of Asians (*p* = 0.001) [33]. A meta-analysis estimated that the risk of developing GDM increases with weight gain and is not affected by location; compared to the control group, the risk of developing GDM is approximately two, four, and eight times higher in overweight, obese, and extremely obese women, respectively [34].

Several studies have highlighted that women who have a positive family history of diabetes, particularly among first-degree relatives, are at an elevated risk of developing gestational diabetes and type 2 diabetes [35]. These conditions arise from a complex interplay between genetic predisposition and environmental influences. A comprehensive systematic review and meta-analysis have revealed that specific minor alleles of nine single-nucleotide polymorphisms (SNPs) within seven distinct genes, including rs7903146 (in TCF7L2), rs12255372 (in TCF7L2), rs1799884 (-30G/A, in GCK), and rs5219 (E23K, in KCNJ11), which play pivotal roles in regulating insulin secretion, are significantly associated with an elevated risk of gestational diabetes mellitus (GDM) [36]. Advanced maternal age has been associated with an elevated risk of GDM. A significant prospective study revealed that women who are over 40 years old exhibit more than a twofold increase in the risk of GDM compared to women who are younger than 30 years old (prevalence of 9.8% versus 4.1%, respectively) [37]. Furthermore, the risk of GDM showed a linear relationship with maternal age [38].Our research findings also demonstrated that both age and family history are independent risk factors for PCOS.

Testosterone (T), a vital androgenic hormone found in the bloodstream, is primarily synthesized by the ovaries. However, in the context of Polycystic Ovary Syndrome (PCOS) patients, an excessive production of testosterone disrupts proper ovary development and leads to irregular ovulation, ultimately resulting in infertility. Thus, accurate measurement of blood testosterone levels serves as a crucial diagnostic parameter for the precise identification of PCOS [39]. Several studies have highlighted that elevated levels of testosterone and decreased sex hormone-binding globulin (SHBG) are independent risk factors for gestational diabetes mellitus (GDM) in patients with PCOS. Possible underlying mechanisms could involve disruptions in hormonal secretion during pregnancy, reduced insulin sensitivity, and direct stimulation of the ovaries, leading to heightened androgen levels [40, 41]. The univariate analysis in our study revealed a significant difference in T levels between the two groups, but the results of the multivariate analysis did not show any statistical significance. This discrepancy could be attributed to the limited sample size and the confounding effects of other factors.

Recently, much attention has been paid to the role of other hormone factors in the development of GDM. The prediction indices included Follicle-Stimulating Hormone(FSH), Luteinizing Hormone(LH), and Thyroid peroxidase antibody (TPA). The prediction time includes the first and second trimester of pregnancy, but there is no simple and practical prediction index with high sensitivity and specificity. Therefore, we should consider other parameters for predicting GDM in women with PCOS.

We conclude that insulin, age, TC, HbA1C, and family history were effective risk predictors for GDM in women with PCOS in the first trimester. Our analysis was limited because all data used for analysis were obtained from a single site, which may have impaired our analysis. A multicenter validation using a large number of patients may produce results that are more generalizable to the broader population.

## Data Availability

The datasets analyzed during the current study are not publicly available due to the metadata containing information that could compromise the patients but are available from the corresponding author on reasonable request.
